# Developing High-Resolution Population and Settlement Data for Impactful Malaria Interventions in Zambia

**DOI:** 10.1155/2022/2941013

**Published:** 2022-09-27

**Authors:** Olena Borkovska, Derek Pollard, Busiku Hamainza, Emmanuel Kooma, Silvia Renn, Jolynn Schmidt, Hasim Engin, Matthew Heaton, John M Miller, Paul Psychas, Christina Riley, Annie Martin, James Nyirenda, Frazer Bwalya, Anna Winters, Corey Sobel

**Affiliations:** ^1^Geo-Referenced Infrastructure and Demographic Data for Development (GRID3), Center for International Earth Science Information Network (CIESIN), Columbia Climate School, New York, USA; ^2^Akros, Lusaka, Zambia; ^3^National Malaria Elimination Program, Lusaka, Zambia; ^4^Geo-Referenced Infrastructure and Demographic Data for Development GRID3, African Sun Consulting, Lusaka, Zambia; ^5^PATH Malaria Control And Elimination Partnership in Africa (MACEPA), Lusaka, Zambia; ^6^U.S. President's Malaria Initiative, U.S. Centers for Disease Control and Prevention, Lusaka, Zambia

## Abstract

Foundational high-resolution geospatial data products for population, settlements, infrastructure, and boundaries may greatly enhance the efficient planning of resource allocation during health sector interventions. To ensure the relevance and sustainability of such products, government partners must be involved from the beginning in their creation, improvement, and/or management, so they can be successfully applied to public health campaigns, such as malaria control and prevention. As an example, Zambia had an ambitious strategy of reaching the entire population with malaria vector control campaigns by late 2020 or early 2021, but they lacked the requisite accurate and up-to-date data on infrastructure and population distribution. To address this gap, the Geo-Referenced Infrastructure and Demographic Data for Development (GRID3) program, Akros, and other partners developed maps and planning templates to aid Zambia's National Malaria Elimination Program (NMEP) in operationalizing its strategy.

## 1. Introduction

Zambia is a highly endemic malaria country and is among the 20 countries reporting the highest malaria incidence and mortality globally, with the entire population considered at risk of malaria transmission. [1] The government of the Republic of Zambia had set a goal of eliminating local malaria infection and disease in Zambia by 2021. [2].

The country's Ministry of Health relies on a range of interventions, including community-based surveillance and vector control measures, to fight the disease. Since 2017, the National Malaria Elimination Program (NMEP) has deployed indoor residual spraying (IRS) as its primary malaria vector control tool, complemented by distribution of long-lasting insecticidal nets (LLINs) [3]. Maximizing population coverage between these two tools is essential to lessening the high malaria burden; thus, accurately understanding population distribution at a granular level is a key to ensuring enough resources reach each district and health facility. [4] Each year, campaign planning processes determine, where IRS will be applied, and every two to three years, where LLINs will be distributed.

NMEP had the ambitious strategy of conducting a combined IRS and LLIN campaign to reach the full population with vector control by late 2020 or 2021. The government's “mosaic approach” aimed to conduct IRS campaigns in prioritized zones of all districts, with the mass distribution of LLINs to fill gaps at sub-district level. At the time of the 2020 campaign, Zambia administrative division constituted 10 provinces and 116 districts. According to longstanding Zambian practice, the selection of settlements for IRS within districts was based on criteria of structure density, suitability of construction materials, accessibility, and other aspects of operational feasibility. To ensure every settlement was covered with at least one vector control intervention, joint IRS/LLIN micro planning sessions were conducted in each district nationwide. However, in the beginning of 2020 the required accurate and up-to-date key data on residential structure counts and population distribution, which determine IRS and LLIN resource needs, respectively, were still lacking.

Foundational high-resolution geospatial data products are valuable additions to the efficient planning of resource allocation during critical health sector interventions such as malaria control [5]. To ensure the relevance, usability, and sustainability of these products, government partners must be involved from the beginning in programs to create, improve, and/or manage data, placing a premium on close cooperation with government stakeholders, as well as on capacity strengthening efforts. [6] With that in mind, Geo-Referenced Infrastructure and Demographic Data for Development (GRID3), Akros, Program for Appropriate Technology in Health (PATH) and the President's Malaria Initiative (PMI) contributed to a multifaceted initiative supporting the Zambian government's campaign to maximize access to vector control. This group of partners with unique expertise contributed toward designing adaptable and relevant geospatial solutions to aid the efforts of NMEP with planning for 2020 malaria vector control campaigns. GRID3's multi-year engagement in Zambia and experience in working with the Zambia government to generate, validate, and use geospatial data on population, settlements, infrastructure, and boundaries, ensured access to relevant data required for the development of micro planning maps. Akros has extensive technical experience supporting Zambia's malaria intervention decision workflows with the MOH NMEP, through implementing geospatial and digital tools over the last 10 years. One such tool is Reveal (https://revealprecision.com/), a digital open-source decision support tool. Reveal allows for verifying structure-level data and uses geospatial data products, including those from GRID3, to precisely track the delivery of in-field activities to ensure complete and accurate coverage.

This paper describes the collaborative process of the partnership's ability to: (1) generate high-resolution geospatial data to enhance the efficient planning of resource allocation; (2) incorporate such data to create a planning map template; and (3) implement a map template during micro planning sessions and generate final map products for all districts; and use the Reveal tool, an open-source digital spatial intelligence platform, in a subset of districts to support the planning, execution, and monitoring of intervention activities. The development of these geospatial data products supported more targeted service delivery, a better understanding of health interventions achieved, partial digitization of campaigns, and communication and harmonization of geospatial data across the government and its partners.

## 2. Materials and Methods

### 2.1. Generating Data for Maps

In April of 2020, the partners listed above initiated a collaborative process led by the Zambia's NMEP to utilize data produced by GRID3 to create micro planning maps for the vector control campaigns in all 116 districts across the 10 provinces. Data utilized for the production of user-friendly planning maps included the high-resolution gridded population estimates, settlement extents showing delineation of settled areas nationwide, and the number of residential structures, settlement names, and administrative district boundaries, as well as locations of landmarks such as health facilities and schools. These detailed maps were used to (1) ensure that all settlements and their populations within a given district were accounted for in service delivery as per the NMEP strategic plan, (2) ensure that there were enough vector control resources (e.g., insecticides, pumps and PPE for IRS, and LLINs personnel) to reach all settlements targeted by either IRS or LLIN across all districts, (3) to improve understanding of the accuracy of reported coverage, and (4) to communicate and harmonize geospatial data across the government and its partners. The following sections describe the production of geospatial data inputs that were used in the creation of the maps.

#### 2.1.1. Population Estimates

In partnership with Zambia Statistics Agency (ZamStats), formerly the Central Statistical Office), the GRID3 Zambia team produced high-resolution population estimates that rely on household surveys to model population in a Bayesian framework at a spatial resolution of approximately 100m by 100m [7]. GRID3 Zambia produced these gridded population estimates using a bottom-up modeling approach as described by Dooley et al. [8] and similar to those previously described by Leasure et al. [9] and Boo et al. [10]. Innovations of the GRID3 Zambia model include the use of building footprints derived from high-resolution satellite imagery and population data for validation of modeled estimates that were solely collected by the government of Zambia. Because of availability of recently collected survey data by ZamStats and the use of advanced location recording techniques, GRID3 was able to use the survey population counts for refining population modeling. Using existing field-collected data for this purpose meant that no extra fieldwork was needed to carry out the work.

#### 2.1.2. Health Facilities and Schools

GRID3 obtained existing health facility location data from government sources, including the Ministry of Health (MoH) and ZamStats, to assess coverage and produce a standardized health facility dataset “NSDI Zambia Operational Health Facility Points and Names, Version 01 (Beta)” [11]. Accurately locating schools on the maps were considered important for providing landmarks for user orientation. The input school data to produce “NSDI Zambia Operational School Points and Names, Version 01 (Beta)” [12], were collected by the Ministry of General Education (MoGE), ZamStats, and the Ministry of Water Development Sanitation and Environmental Protection (MWDSEP) between 2010 and 2018. The health facility and school names were standardized for consistency and ease of labeling, with type and subtype attributes added to distinguish among various health facility and school types. Location attributes were also added to the datasets to note within which province and district each point is located.

#### 2.1.3. Settlement Extents and Settlement Names

Settlement extents are polygons representing areas where a human settlement is likely, based on the presence of buildings detected in satellite imagery. Settlement extents that show population distribution are a key data input for micro planning maps. [13] Prior to this initiative, a precise rendering of Zambia's population distribution had not been produced; the inclusion of these extents represents an important evolution in the country's geospatial data foundation. In addition to serving as one of the most accurate renderings of the country's population distribution, these extents can also help to reduce survey costs (as they eliminate the need for field mapping to be conducted nationwide).

Settlement extents are not meant to represent the boundaries of an administrative unit or locality. A single settlement extent may be made up of multiple localities, especially in urban areas. Both the settlements' extents and classification are derived solely from building footprints extracted from high-resolution imagery [14]. Data analysis and processing were achieved entirely using Esri's ArcGIS software (pro version 2.7.3), its native module arcpy, and open-source python library pandas 1.3.0.

The names and GPS point location of settlement names were developed by compiling existing data sources from the government institutions; settlement names were extracted from a 2010 government mapping exercise, during which points of interest (POIs) nationwide were collected by ZamStats. The settlement points were also compared against nearly 12,000 settlement points from the Ministry of Water Development, Sanitation, and Environmental Protection. All available sources were compiled, merged into one layer, and compared against settlement extents derived from the building footprints to ensure a point fell within a settled area [15].

#### 2.1.4. Settlement Residential Structure Estimates

Building densities refer to the total number of building points, or structures of all types, within the settlement. To estimate the number of eligible structures for IRS planning, a predictive statistical model was built and applied to the building density to produce a residential structure estimate. Using QGIS, Stata, and *R*, this residential structure estimation model was created using GRID3 settlement structure counts and compared against field-verified malaria implementation data collected through the Reveal platform in 2019 and 2020. Predictive factors of the number of residential structures are primarily related to settlement size and structure density, with some regional geographic differences. The model was rebuilt and validated with 2020 field-verified data reporting an absolute total predictive accuracy of 20% of the true value (i.e., ±10%), with the accuracy of the prediction increasing as settlement size decreased. The average absolute difference between predicted and actual residential structure estimates was about one-to-two structures, except for settlements above 400 structures which comprised less than 1% of settlements in the field-verified dataset.

### 2.2. Developing a Map Template

To ensure maps are actively used by decision-makers, a map template was developed in consultation with implementors (chiefly, the MOH at the district level and VectorLink) to aid districts in micro planning. The map templates were designed to: (1) render easier distinction of spatial populations and settlements; (2) maintain legibility of map content when subdividing the full extent of Zambia into regularly-proportioned index grid cells; (3) allow replication, scaling, and use for all 116 districts and for future intervention campaigns. A flexible grid system was devised using harmonized district boundaries to generate the index study areas and nested reference grid cells. Reference grids were used to summarize residential building and population counts, and to create corresponding alphanumeric settlement names for organizational purposes (Figure 1).

#### 2.2.1. The Index Grid

Each of Zambia's 116 districts was subdivided into a 289-cell static Index Grid using the output of the ArcGIS Grid Index Features Tool as a baseline. This index grid was used to determine the extent of each map page driven by ArcGIS Pro's Map Series feature. Each page was locked to a 4 : 3 (landscape) or 3 : 4 (portrait) aspect to ensure it could be subdivided into equal-area grid cells. Each baseline index cell was 60 km × 80 km, adjusted as necessary depending on the size and shape of the district they subdivided. In order to prevent symbols and labels from being too small to read at A0 printed page size, maps were given a hard constraint of 1 : 1,000,000 scales. After the final index grid was created and cleaned, each page was subdivided into 12 regular, equal-area reference cells.

#### 2.2.2. The Reference Grid

The index grid output, detailed abovementioned, was then used as an input for the second iteration of Grid Index Features. Sub setting each map into a series of nested grids was useful in two ways. First, nested grids allowed for tabular summaries of grid features to be included on the maps. Using the included tables, users can parse, at a glance, summary statistics and how they relate to different subdivisions of the map document. Whereas index grid pages may depict overlapping areas, reference grid cells were clipped to an exclusive study area, which subtracted all nonrelevant space from the analysis. This ensured that summary statistics related to each grid cell were not double-counted among map pages. The sum of these grid cells was used to calculate per-page summary statistics, and the sum of those sums was in turn used to calculate per-district summaries. Tables summarize settlement counts, full district totals, map page totals, and reference grid cell totals, as well as per-settlement summaries of population and building count. Second, dividing each district into low-level grid cells allowed for the creation of an easily distinguishable unique identifier scheme for every settlement that had 25 or more residential structures within it. Each of the 12 reference grid cells contained its own alphanumeric code (A1, B2, C3, etc.) to which settlements were assigned, sorted by latitude, and numbered sequentially [16].

#### 2.2.3. Map Design

Maps were designed to be viewed at A0 poster size, which gave wide latitude to the level of detail that could be included on the map page. Because of the large volume and density of information necessary to include on the map templates for operations planning, readers' attention needed to be managed hierarchically. To keep the information displayed on the maps efficiently [17], the prioritized data included were: (1) settlement location, (2) settlement size threshold differentiating larger settlements (defined as 25 or more residential structures) and smaller settlements (fewer than 25 structures), and (3) estimated population and residential building counts. All other information (boundaries, road networks, health infrastructure, etc.) was ancillary and to be used to orient the user in space. Foreground/background separation was established primarily through color and transparency [17]. Settlements were depicted in fluorescents. Larger settlements were outlined in cyan, with fills of yellow and orange-red population ramps. Far smaller but more numerous smaller settlements were outlined in magenta, with slightly transparent magenta fills. Settlement types were further distinguished by their labels: large settlements each had text box callouts, describing their alphanumeric name, estimated population sum, and estimated residential building count. In the interest of reducing page crowding, small settlements were labeled only with their building count, italicized in the center of each polygon [18]. A semi-transparent masking overlay was applied to deprioritize space outside of the active sub-district study area while preserving the user's sense of place within a larger context. Point of interest symbols and labels were preserved but de-emphasized by converting to grayscale, reducing size, and/or reducing opacity.

A simple terrain hillside was used as the template' s embedded base map in order to provide additional spatial context and inform users of natural barriers to further facilitate planning exercises. Road networks and water features from OpenStreetMaps (https://www.openstreetmap.org) were similarly incorporated. Special consideration had to be taken to avoid using hosted base maps with integrated and possibly outdated administrative boundaries, as GRID3 worked closely with the Office of the Surveyor General, Ministry of Local Government, Electoral Commission of Zambia, and Zambia Statistics Agency in order to provide the most accurate and up-to-date boundaries available [19].

#### 2.2.4. Map Piloting

To enhance the map's usability and alignment with district planning needs during district-level micro planning activities, prior to their finalization, sample maps and training materials were generated and piloted in the following three districts to collect feedback from provincial and district managers: Kasama District in Northern Province, Mwansabombwe District in Luapula Province, and Solwezi District in North-Western Province. These three districts were selected because of their diverse contexts and distribution across different provinces. They were all within PMI operational areas to ensure VectorLink teams could readily provide piloting logistical support. Participants were primarily the same District Health Officers (DHOs), Provincial and National staff, who would later be involved in the district-level IRS and ITN campaign micro planning activities for which these mapping tools were being designed. The NMEP vector control team lead this piloting process, with support from Akros and VectorLink, organizing online map use training and feedback sessions. Each district was also reached out separately to maximize feedback on suggested changes.

## 3. Results

Feedback from the DHO staff in these three districts during the piloting process suggested that the inclusion of maps along withuser guiding documents to enhance resource allocation decisions during micro planning activities and to guide deployment was highly valued. Suggested changes gathered led to map design changes that were incorporated into the final maps, user guides, and training materials. Having the NMEP vector control team lead these feedback sessions ensured the district participants that their efforts would help improve the NMEP micro planning outcomes and thus led to quick highly engaged feedback. During the actual campaign micro planning sessions in Western Province, positive qualitative feedback was collected through six survey questions, collecting responses from 25 participants representing all 16 districts in that province. Survey participants indicated that the maps and population tables were very useful in demonstrating distribution of settlements across the district, how large they were, and how easy/difficult they are to reach (all of which informed prioritization of where IRS versus LLIN resources would be applied). It was reported the process of demarcation and filling out the planning templates using information from the maps was easy to follow in order to calculate the total number of structures targeted for IRS and the population targeted for LLINs. This helped managers to understand if the resource allocation provided by the national level was over estimated (which potentially wastes resources) or under estimated (which means some settlements are excluded).

Some feedback from provincial and district managers indicated the need for minor changes to the planning templates. For example, a primary challenge experienced during the pilot was the exclusion of health facility catchment area (HFCA) boundaries on the map. This made it difficult to understand which settlements, and therefore population and structure counts, fell within a specific catchment. Given resource planning and implementation monitoring are required at the catchment level for input into the NMEP DHIS2 health information system, being able to accurately map settlements to the correct catchment is very important. Another limitation was that accurate catchment boundaries were not available and adding modelled ones would have led to inaccurate health facility level planning outputs. In addition, the pilot district teams noted the difficulty in understanding the village or area to which each settlement belonged, as there were not enough features (points of interest data) on the GRID3 map to provide “locational context” to the user. Lastly, once targeted demarcations were made on the maps, the counting of the population within the smaller settlements, less than 25 structures, was error-prone, particularly when there were many settlements within the demarcated area.

This specific feedback was used to refocus the purpose of the maps from providing health facility planning outputs to providing district-level structure counts targeted for IRS and population counts targeted for LLINs. These counts could then be compared to the district-level resources made available to determine if enough resources were available to cover the entire district and to encourage districts to advocate for more resources (if required). The main map template changes included the addition of village names, schools, water bodies, roads, railways, and forest reserves to help orient users in the field. Index grids were also added to the map and aggregation tables, to help divide the district, encouraging smaller demarcations and easier counting of population and structures on the map. However, as previously mentioned, time did not permit the incorporation of HFCA boundaries; these were added after the 2020 campaigns as an enhancement for future use.

Once the map template was finalized, maps were generated from the template for all 116 districts (289 maps at A0 page size) and disseminated through government micro planning workshops. NMEP conducted the annual planning processes at the national level via the NMEP Vector Control Technical Working Group and at the district level through three-day micro planning workshops held in each province, during which it was determined where IRS would be applied and where bednets would be distributed. During the district micro planning process, key staff from the district level vector control teams, guided by provincial and national malaria trainers, used the printed A0 maps to understand the population and residential structure distribution across their district. With an understanding of the malaria burden and operational constraints across their district, they drew IRS as well as LLIN targeting demarcations on the maps to help inform prioritization and resource allocation decisions at sub-district level. Through understanding the location and size of each settlement within their district in relation to health facility sites, access routes, deployment sites, and resource availability for each intervention, map use during micro planning informed decisions on where each intervention (IRS or LLINs) should be implemented. The process outcomes highlighted any settlements that had been left out and if available resources were likely to be enough to cover all the structures within settlements demarcated for IRS and the population within settlements demarcated for LLIN's. In addition, the maps aided in deployment planning for their vector control interventions by clearly demarcating that settlements were planned to receive IRS versus LLIN' s. While the micro planning map user guide document encouraged discussion to resolve any gaps, any resulting changes were not formally documented.  Figure 2 shows an example of a final district map produced by GRID3 for Mwansabombwe District, Luapula Province, while Figure 2 shows a detailed view of the map.

Once the IRS targeted areas were demarcated on the paper maps, the targeting demarcations were digitized and used within Reveal to support IRS implementation in 21 districts across the Western and Southern provinces. Reveal displayed the geospatial data on field teams' mobile devices, navigating them to those settlements that were targeted during micro planning and providing a high-resolution satellite imagery view of the village they are in to understand the distribution of structures within the area. The Reveal dashboards provided the digitized campaign “denominator” to accurately monitor and calculate IRS coverage as daily spray reports came in. In 7 of these 21 districts, Reveal technicians were embedded in the spray teams and marked in real time whether structures were found and sprayed. The teams relied on Reveal to (1) navigate to target areas and houses, (2) track whether GRID3 settlements targeted during planning were actually visited in the field, and (3) track health facility catchment level coverage against the GRID3 population denominator. The rest of the 102 districts relied on paper-based maps.

## 4. Discussion

This paper outlined the process applied to create map products that served to inform macro- and micro-level planning of malaria campaigns in Zambia. The information gained through the 3-district pilot of these products informed the further scale and deployment of maps across 116 districts in Zambia. Previous to these efforts, household mapping had been undertaken, both through the use of GPS units (initially) and later through desk-top digitization of satellite imagery at the household level [20]. The approach described herein of producing population and structure data at the settlement level offers an option for efficient delivery of map products for planning processes--future work will further compare this approach with existing methods (such as enumeration of satellite imagery).

The maps used during the micro planning demarcation process, to understand population down to settlement level, included modeled population counts as opposed to official census population data that were only available down to district level. The modeled population dataset provided the Government of Zambia and partners with estimates of the population across the country, at a very high resolution and based on recent enumeration data. The dataset provides a detailed picture of where people in Zambia live, with the gridded nature of the dataset providing flexibility in calculating the population per settled area. This level of detail allowed the government to effectively plan and implement malaria activities at the sub-administrative level.

Delivery of map products occurred both in paper-based format and also through the digital platform, Reveal. A forthcoming publication highlights the process for operationalizing these products. The integration of the GRID3 product with Reveal highlights the potential for end-to-end digitization of the campaign planning and delivery process, applicable to the campaign and also routine health service delivery (e.g., ICCM). GRID3's map product provides base maps of population data, while Reveal operationalizes these base maps to support planning and also the in-field use of the digital maps to guide field teams and monitor their progress in campaign delivery/coverage. Given this recent work, the ongoing and future application of GRID3 products looks promising for the delivery of various health campaigns (including malaria, neglected tropical diseases, vaccination, and community health). Lessons learned during the 2020 implementation informed changes to the now-complete 2021 maps. For example, in 2021, the MoH and funding partners (including PMI and PATH) requested these planning maps be used again across the country, not only to support vector control planning for malaria but also to support other health sector programs (such as routine immunizations and COVID-19 micro planning support).

Throughout the process of generating map products for malaria campaigns in Zambia, several limitations have been observed. One of the key limitations was the absence of health facility catchment area boundaries, which are field mapped and endorsed by district health staff and available in a digital format. Given that health interventions in Zambia are planned down to the catchment level, the absence of such operational level boundaries made it difficult for district health teams to assess the need for resources at the unit of geography at which the operational provisions often take place. Health facility catchment area boundaries were later mapped, in early 2021, and included in the micro planning maps to address this limitation in time for the 2021 vector control planning activities.

Despite the presumed accuracy of the enumeration data from surveyed locations, used as an input to GRID3's model, modeled datasets remain statistical estimates which are not a replacement for robust, complete enumeration [20]. However, given the opportunity to quickly scale maps for planning purposes through the GRID3 model, this methodology is worth continued pursuit, with an option for fine-scale enumeration to focal areas if needed. It is worth noting that locations of settlement extents have not been field-verified nationwide, thus settlement extents that are rural and have an estimated population of less than five people are subject to higher uncertainty. The future release of settlement extents will be improved to ensure improved validation procedures to decrease the number of false positives.

## 5. Conclusion

The need for accurate, up-to-date, and accessible geographic data on population distribution is a fundamental requirement necessary to deliver health services to everyone. Without those data, country planning processes and implementation of health services are hindered. This paper summarizes the successful development of paper-based maps incorporating GRID3 data, through a consultative partnership among the MOH, NMEP, and partners. The approach taken here showcases how maps may be developed at scale for micro planning processes to plan for and improve large-scale health campaigns; in this case, IRS and LLINs for malaria control. Future research would be useful to describe the potential cost-savings achieved through the use of geo-enabled planning processes, which is believed to be significant.

## Figures and Tables

**Figure 1:** Grid system developed using district boundaries (left) for production of the index study area (center) and nested reference cells (right).

**Figure 2:** District map: An example of a map created with the dynamic map template.

## Data Availability

The data used for production of the microplanning maps have been deposited in the GRID3 repository (https://data.grid3.org/), Columbia Academic Commons (https://academiccommons.columbia.edu) and the WorldPop Open Population Repository (WOPR) (https://wopr.worldpop.org/?/Population). The settlement extents and number of structure counts are derivative works from Digitize Africa, powered by Maxar Technologies, Inc. and Ecopia Tech Corporation. By using the derived map, you agree to be bound to the terms of use and conditions from the Ecopia Digitize Africa Data Humanitarian License v1.0, Annex 2.
